The article "Clinical Study on Efficiency of Using Traditional Direct Bonding or OrthGuide Computer-Aided Indirect Bonding in Orthodontic Patients" was published in 2022. Journal: Dis Markers.

# Clinical Study on Efficiency of Using Traditional Direct Bonding or OrthGuide Computer-Aided Indirect Bonding in Orthodontic Patients

**DOI:** 10.1155/2022/9965190

**Published:** 2022-09-29

**Authors:** Min Wang, Xing Shi, Wei-Pu Cheng, Fei-Hu Ma, Si-Miao Cheng, Xuan Kang

**Affiliations:** ^1^RYTIME Dental, Beijing 100000, China; ^2^Shenzhen Becoming Digital Dental Co., Ltd., Shenzhen 518000, China

## Abstract

**Objective:**

This study aims to clinically investigate and compare the therapeutic effects and treatment cycle between traditional direct bonding and OrthGuide computer-aided indirect bonding in orthodontic treatment.

**Methods:**

Forty patients treated at the Department of Orthodontics, Beijing Rytime Dental Hospital between July 1, 2016, and December 31, 2019, were included. The patients were divided into a control group (*n* = 20, traditional direct bonding) and a test group (*n* = 20, OrthGuide computer-aided indirect bonding). The American Board of Orthodontics (ABO) measurement was performed on patients using Uceph cephalometric analysis software to compare intragroup and intergroup differences, and the treatment cycles of all patients were recorded.

**Results:**

After treatment, U1-NA (mm), ∠U1-SN (°), LL-EP (mm), and UL-EP (mm) in the control group were significantly lower than before treatment, and there was no significant difference in other ABO measurement indexes, while the test group showed no marked difference in all ABO measurements between pre- and posttreatment. Further, intergroup comparison showed no significant difference in ABO measurements in pre- and posttreatment between the two groups. The test group had a shorter treatment cycle than the control group, with an average treatment cycle of 21.20 ± 7.14 months in the control group and 17.17 ± 4.16 months in the test group.

**Conclusion:**

There was no significant difference in the therapeutic effects between the direct and indirect bonding techniques. However, OrthGuide computer-assisted indirect bonding demonstrated a significantly shorter treatment cycle and might be more efficient than traditional direct bonding.

## 1. Introduction

Orthodontic treatment is the correction of dentition and facial profile in patients with various types of malocclusion [1, 2]. About 50 years ago, Andrews invented the world's first straight wire appliance to simplify clinical procedures and shorten treatment duration. Additionally, the straight wire appliance greatly reduced the reciprocating movement of teeth due to mistakes in edgewise archwire bending [3, 4].

With the innovation of technology and the rapid development of the computer industry, more and more clinicians and researchers are combining orthodontics with computer technology, and several breakthroughs have been achieved. The direct bonding of straight wire brackets depends on clinicians' experience and dentition observation to a certain extent. As a result, bracket bonding may be of limited accuracy, easily leading to the reciprocating movement of teeth before the end of treatment, increased the number of follow-up visits, and prolonged treatment duration. The main objective of an orthodontist is to provide high-quality treatment within a reasonable timeframe. To achieve this, researchers have developed several techniques to improve the quality of orthodontic treatment by using new technologies such as indirect bonding and custom brackets and arches or computer-aided design software.

The article "Clinical Study on Efficiency of Using Traditional Direct Bonding or OrthGuide Computer-Aided Indirect Bonding in Orthodontic Patients" was published in 2022. Journal: Dis Markers.

Indirect bonding refers to a technique in which the bracket position is planned by a computer, and the corresponding guide plates are printed. This technique can accurately bond the bracket, improve the orthodontic efficiency, and realize the accurate and rapid movement of the teeth to a desired location [5, 6]. In addition, the computer can simulate the process and effects of orthodontic treatment, helping dentists to understand the feasibility of the orthodontic plans. In this regard, OrthGuide computer-aided indirect bonding technique can achieve accurate bracket bonding and simplify orthodontic operation, thus improving the stability of orthodontic treatment and shortening the orthodontic cycle [7].

The aim of this study was to compare the results and treatment cycles between traditional direct bonding and OrthGuide computer-aided indirect bonding in orthodontic treatment to provide a relevant theoretical basis that could help clinicians select more appropriate fixed orthodontic appliances.

## 2. Materials and Methods

### 2.1. Study Subjects

Forty patients who received orthodontic treatment at the Department of Orthodontics, Beijing Rytime Dental Hospital, from July 1, 2016, to December 31, 2019, were selected. They were divided into a control group (*n* = 20, traditional direct bonding) and a test group (*n* = 20, OrthGuide computer-aided indirect bonding) according to their wishes. All patients received orthodontic treatment from the same professional dentist. This study was approved by the Ethics Committee of Beijing Rytime Dental Hospital, and patients (or parents or guardians of minor patients) signed informed consent before the treatment. The study inclusion criteria were (1) healthy patients from both sexes aged 12-55 years; (2) no previous orthodontic treatment; (3) presence of tooth displacement; (4) individual normal occlusion after orthodontics; and (5) presence of minimum four permanent teeth (except molars) to be bonded in each of the four quadrants (thus extraction or nonextraction cases) and all teeth fully erupted. Patients were excluded if they had (1) moderate or severe periodontitis; (2) severe temporomandibular disorders; (3) systemic diseases such as coagulopathy; (4) severe jaw deformity; (5) teeth presenting active caries, fluorosis or hypoplasia of enamel, restorations, or fractures of the surfaces to be bonded; and (6) abnormalities in crown morphology of the teeth to be bonded.

The article "Clinical Study on Efficiency of Using Traditional Direct Bonding or OrthGuide Computer-Aided Indirect Bonding in Orthodontic Patients" was published in 2022. Journal: Dis Markers.

### 2.2. Grouping and Treatment

The control group received a straight wire appliance with traditional direct bonding of brackets. The test group used DamenQ self-ligating brackets (Ormco, USA) combined with OrthGuide computer-aided indirect bonding. The patients' dentition was aligned according to a conventional orthodontic process to level and align the teeth, close the space, slightly and finely adjust the occlusion, and achieve individual normal occlusion.

### 2.3. American Board of Orthodontics (ABO) Measurement

Before and after orthodontic treatment, the lateral cephalogram was taken by the same radiologist. The images were obtained using a dental X-ray digital tomography equipment (KaVo Sybron Dental [Shanghai], China, 220 V), with 90 kV, 13 mA, and 16 s scanning time conditions. The measurement of the American Board of Orthodontics (ABO) was performed using the UCeph 4.4.2 software (Yaxun Technology (Chengdu) Co., Ltd., China), and the obtained data were recorded. The measured items were as follows: (1) sagittal direction: ∠SNA (°), ∠SNB (°), ∠ANB (°), U1-NA (mm), ∠ U1-SN (°), L1-NB (mm), ∠ L1-MP (°), LL-EP (mm), and UL-EP (mm) and (2) vertical direction: ∠SN-MP (°) and ∠MP-FH (°).

### 2.4. Statistical Analysis

All data were analyzed using the SPSS 22.0 statistical software. Measurement data were first tested for normality. ABO measurement results that failed to meet the normal distribution, so the Kruskal-Wallis test was used for analysis. The paired *t*-test was used for orthodontic treatment cycles that met the normal distribution. *P* < 0.05 was considered statistically significant.

## 3. Results

### 3.1. General Clinical Information

A total of 40 patients were eligible for this study. There were 20 (5 males and 15 females) patients in the control group, including 5 cases of Angle's class I, 13 cases of Angle's class II, and 2 cases of Angle's class III. They were 12–29 years old and had a mean age of 18.75 ± 6.50 years. There were 20 (3 males and 17 females) patients in the test group, including 6 cases of Angle's class I malocclusion, 13 cases of Angle's class II malocclusion, and 1 case of Angle's class III malocclusion. The patients in the test group were 12 –55 years old and had a mean age of 21.35 ± 10.99 years. There was no significant difference in pretreatment cephalometric data between the two groups (*P* > 0.05, Table 1), indicating that the two groups were comparable.

The article "Clinical Study on Efficiency of Using Traditional Direct Bonding or OrthGuide Computer-Aided Indirect Bonding in Orthodontic Patients" was published in 2022. Journal: Dis Markers.

### 3.2. Intragroup Comparison of American Board of Orthodontics (ABO) Measurements in Pre- and Posttreatment

All patients achieved individual normal occlusion after treatment. No significant difference was found before and after treatment in the test group (*P* > 0.05, Table 2). Comparatively, in the control group, the sagittal parameters UI-NA (mm), ∠U1-SN (°), LL-EP (mm), and UL-EP (mm) after treatment were significantly lower than those before treatment (*P* < 0.05, Table 3), but no marked differences were observed in other measurement items (*P* > 0.05).

### 3.3. Intergroup Comparison of American Board of Orthodontics (ABO) Measurements in Posttreatment

ABO measurements showed no significant posttreatment difference between the two groups (*P* > 0.05), indicating that direct bonding and OrthGuide computer-aided indirect bonding had similar orthodontic correction results (Table 4).

### 3.4. Comparison of Orthodontic Correction Cycles between the Two Groups

The time span from initial diagnosis to the end of treatment was recorded as the treatment cycle of each patient. The comparison results showed that the overall treatment cycle of the test group was significantly shorter than the control group (*P* < 0.05, Table 5).

## 4. Discussion

Orthodontic treatment is usually efficient, functional, stable, and comfortable. Therefore, the goal of orthodontists is to achieve individualized and accurate bonding of brackets onto the labial surfaces of each tooth, thus ensuring a more efficient and stable movement of teeth [8–11]. Direct bonding of orthodontic brackets onto teeth can be achieved with the naked eyes of orthodontists, while indirect bonding is created by a 3D model of teeth with the aid of an OrthGuide computer [5, 12–14]. The latter ensures more accurate positioning of brackets and more efficient tooth movement. Shpack et al. [15] and Bozelli et al. [16] reported no statistical difference in the length of chairside operation time between direct and indirect bonding. However, the time taken might be related to the clinician's operation proficiency; i.e., more skilled doctors usually have shorter clinical chairside operation time.

Although the accuracy of bracket positioning has not been further investigated in our study, some scholars have reported relevant results. Chen et al. [17] showed that the registration accuracy of a 3D maxillodental model could reach 0.1-0.4 mm, and the actual position of the bracket orientated by indirect bonding trays was nearly identical to the virtual position by computer simulation. Qi et al. [18] investigated the clinical effects of digital indirect bonding and found that this technique could make bracket bonding more accurate and make the height of the marginal ridge of the posterior teeth more consistent.

The article "Clinical Study on Efficiency of Using Traditional Direct Bonding or OrthGuide Computer-Aided Indirect Bonding in Orthodontic Patients" was published in 2022. Journal: Dis Markers.

In this present study, no significant difference in ABO measurements was observed between the two groups after orthodontic treatment, but the average treatment cycle of the test group was about 4 months shorter than that of the control group, indicating higher efficiency in the test group. Thus, based on the data, both treatments seemed to be equally effective, but comparatively, OrthGuide was more efficient because it could significantly reduce the time of treatment, thus leading to less pain and hassle for the patients. Brown et al. [7] found that computer-assisted CAD/CAM bonding had the shortest treatment time (13.8 ± 3.4 months) compared with noncomputer-assisted indirect bonding (16.9 ± 4.1 months) and direct bonding (21.9 ± 5.0 months), which was consistent with our findings. After decades of development, computer-assisted indirect bonding has shown advantages in accuracy and tooth movement, for instance, shorter treatment cycles and higher efficiency [19–21]. However, the treatment cycle of this technique depends to some extent on whether the patient is at the peak of growth and development and the type and difficulty of malocclusion. So the conclusion on the treatment cycle after using computer-assisted indirect bonding still needs further investigation.

Our study also had some limitations. First, although the operator and the measurer of the relevant data for both groups of patients were the same physician, no prospective randomization was performed for the enrolled patients. Second, no statistical analysis was performed on the adverse reactions that may occur during and after treatment. Third, there was no further assessment of the cost of the two kinds of orthodontic treatments.

In this era of digitalization, it is expected that CAD/CAM technologies will be improved, and they are going to be more popular due to several benefits, such as their personalized form of orthodontic treatment and being more hygienic. For instance, it was found that stainless steel retainers had higher indicators of bacterial plaque accumulation and gingival inflammation [22], while the smoothness and polish of CAD/CAM retainers caused much less plaque accumulation, thus fewer risks of inflammation [23, 24]. In the future, it would be beneficial to design studies, especially clinical trials with longer follow-up and lower risk of bias, as well as lay more focus on cost to benefit and patients' satisfaction with the use of new technologies to obtain more reliable results about the efficacies and efficiencies of CAD/CAM technologies.

The article "Clinical Study on Efficiency of Using Traditional Direct Bonding or OrthGuide Computer-Aided Indirect Bonding in Orthodontic Patients" was published in 2022. Journal: Dis Markers.

## 5. Conclusion

Compared with traditional direct bonding, OrthGuide computer-aided indirect bonding was associated with a shorter treatment cycle, but there was no significant difference in the effect indexes between the two techniques, suggesting that OrthGuide might be more efficient.

## Figures and Tables

**Table 1:** Comparison of preoperative cephalometric data between the two groups before treatment.

Variables	Control group (*n* = 20)	Test group (*n* = 20)	*P*
∠SNA (°)	80.99 ± 4.30	81.64 ± 2.92	0.55
∠SNB (°)	76.55 ± 4.49	77.69 ± 3.69	0.39
∠SN-MP (°)	37.07 ± 5.65	36.75 ± 5.03	1.00
∠FMA (°)	26.73 ± 4.66	27.78 ± 4.54	0.40
∠ANB (°)	4.44 ± 3.22	3.95 ± 2.11	0.37
UI-NA (mm)	6.20 ± 2.53	5.22 ± 2.34	0.24
∠U1-SN (°)	107.15 ± 9.00	102.01 ± 9.09	0.12
LI-NB (mm)	8.02 ± 4.05	7.46 ± 3.51	0.34
∠IMPA (°)	97.62 ± 11.53	96.88 ± 7.09	0.85
LL-EP (mm)	2.93 ± 2.63	2.90 ± 2.65	0.82
UL-EP (mm)	0.98 ± 2.04	1.26 ± 2.34	0.69

**Table 2:** Comparison of cephalometric data before and after treatment in the test group.

Variables	Before treatment	After treatment	*Z*	*P*
∠SNA (°)	81.64 ± 2.92	81.16 ± 2.75	-0.60	0.55
∠SNB (°)	77.69 ± 3.69	77.69 ± 3.69	-0.26	0.79
∠SN-MP (°)	36.75 ± 5.03	37.04 ± 5.43	-1.10	0.28
∠FMA (°)	27.78 ± 4.54	28.38 ± 4.88	-0.86	0.39
∠ANB (°)	3.95 ± 2.11	3.47 ± 2.28	-1.57	0.12
U1-NA (mm)	5.22 ± 2.34	2.55 ± 4.77	-0.75	0.46
∠U1-SN (°)	102.01 ± 9.09	101.97 ± 9.04	-0.15	0.88
L1-NB (mm)	7.46 ± 3.51	6.56 ± 2.66	-1.21	0.23
∠IMPA (°)	96.88 ± 7.09	93.67 ± 8.25	-1.23	0.22
LL-EP (mm)	2.90 ± 2.65	1.85 ± 2.16	-1.74	0.08
UL-EP (mm)	1.26 ± 2.34	0.56 ± 2.05	-1.87	0.06

**Table 3:** Comparison of cephalometric data before and after treatment in the control group.

Variables	Before treatment	After treatment	*Z*	*P*
∠SNA (°)	80.99 ± 4.30	81.07 ± 4.30	-0.30	0.77
∠SNB (°)	76.55 ± 4.49	76.71 ± 4.57	-1.03	0.31
∠SN-MP (°)	37.07 ± 5.65	37.08 ± 5.80	-0.49	0.63
∠FMA (°)	26.73 ± 4.66	25.92 ± 4.47	-1.59	0.11
∠ANB (°)	4.44 ± 3.22	4.36 ± 2.55	-0.22	0.82
U1-NA (mm)	6.20 ± 2.53	3.85 ± 2.36	-2.80	0.01
∠U1-SN (°)	107.15 ± 9.11	99.82 ± 9.28	-2.65	0.01
L1-NB (mm)	8.02 ± 4.05	6.77 ± 2.54	-1.49	0.14
∠IMPA (°)	97.62 ± 11.53	96.95 ± 8.76	-0.37	0.71
LL-EP (mm)	2.93 ± 2.63	1.74 ± 2.08	-2.17	0.03
UL-EP (mm)	0.98 ± 2.04	−0.07 ± 1.76	-2.69	0.01

**Table 4:** Comparison of cephalometric data between the two groups after treatment.

Variables	Control group	Test group	*Z*	*P*
∠SNA (°)	81.07 ± 4.30	81.16 ± 2.75	-0.28	0.78
∠SNB (°)	76.71 ± 4.57	77.69 ± 3.69	-0.80	0.43
∠SN-MP (°)	37.08 ± 5.80	37.04 ± 5.43	-0.12	0.90
∠FMA (°)	25.92 ± 4.47	28.38 ± 4.88	-0.84	0.40
∠ANB (°)	4.36 ± 2.55	3.47 ± 2.28	-1.54	0.12
U1-NA (mm)	3.85 ± 2.36	2.55 ± 4.77	-1.61	0.11
∠U1-SN (°)	99.82 ± 9.28	101.97 ± 9.04	-1.43	0.15
L1-NB (mm)	6.77 ± 2.54	6.56 ± 2.66	-1.57	0.12
∠IMPA (°)	96.95 ± 8.76	93.67 ± 8.25	-1.16	0.25
LL-EP (mm)	1.74 ± 2.08	1.85 ± 2.16	-1.61	0.11
UL-EP (mm)	−0.07 ± 1.76	0.56 ± 2.05	-0.68	0.50

The article "Clinical Study on Efficiency of Using Traditional Direct Bonding or OrthGuide Computer-Aided Indirect Bonding in Orthodontic Patients" was published in 2022. Journal: Dis Markers.

**Table 5:** Comparison of orthodontic correction cycles between the two groups.

Variables	Control group	Test group
Treatment cycle (month)	21.20 ± 7.14	17.17 ± 4.16
*t*	2.18	
*P*	0.04	

## Data Availability

The data used to support the findings of this study are available from the corresponding author upon request.
